The article "Effects of E-Government Policy on the Management of Healthcare Systems" was retracted in 2023. Reasons: signs of a paper mill; suspected computer-generated content; unreliable results or conclusions; concerns about the data.

# Effects of E-Government Policy on the Management of Healthcare Systems

**DOI:** 10.1155/2022/5736530

**Published:** 2022-01-10

**Authors:** Sarwar Pedawi, Ahmad Alzubi

**Affiliations:** Business Administration Department, Karpas Mediterranean University TRNC, Northern Cyprus, Mersin 10, Turkey

## Abstract

E-government began by addressing the challenges of new technologies by delivering e-services to its citizens and has since evolved to include a growing number of areas, such as citizen communication, macroeconomic projections, budget management, and e-healthcare services. E-government is known as the use of information technology to provide administrative services, communication transactions, information exchange, integration of various electronic systems, and autonomous services between the government and citizens, the government and business environment, and the government and government. This paper discusses the role of E-government policy in healthcare crises during COVID 19. Data collected from 435 employees in the tourism industry of Iraq was used to verify the abovementioned relationships via SPSS macro. The results indicate that E-government policy has a significant effect on healthcare crises; job insecurity negatively predicted healthcare crises. The results revealed that social support moderated the relationship between E-government policy and job insecurity. Results of the study contributed to the theory within this study by demonstrating that employees who enjoy a high level of social support show less job insecurity than those with a low level of social support.

## 1. Introduction

The COVID-19 (Coronavirus Disease-19) pandemic has deeply affected the service industry, particularly tourism. The tourist industry is a significant vehicle for employment creation and economic growth around the world, both directly and indirectly. Strong steps adopted by governments to combat the disease's spread and impact have resulted in hurdles for employees in the sector. Workplace closures, prohibitions on public gatherings, and travel restrictions are examples of such actions. While such measures were intended to slow the spread of the disease, the time spent away from work as a result of the limitations increased the chance of job loss and decreased pay. According to a review of the literature, research has mostly demonstrated the harmful effects of COVID-19 and E-government policies like lockout on health and healthcare problems [1, 2]. According to other research, the e-attempts the government makes to reduce fear of the disease include information about preventative measures, information about the virus, and lockdowns [3]. The E-government, on the other hand, overlooked psychological factors related to people's mental health [4]. From this perspective, it may be argued that additional research is needed to determine the link between E-government policies and healthcare crises, particularly for tourism industry personnel. In addition, little research has been done on how the epidemic has affected employees' healthcare crises. Previous research has focused on specific vulnerable groups such as takeout workers [5], frontline health workers [6, 7], and low-wage migrant workers [3, 6]. These studies were carried out outside of the tourism industry, particularly outside of Iraq, where tourism plays a significant role in the national economy. COVID-19 is also a global issue that has impacted people, societies, organizations, and countries all over the world.

Previous studies have underlined that the fear of job loss is the most critical consequence of E-government policies such as lockdown [8]. Simply put, the measures have made employees in the industry more uncertain and given them a heightened feeling of perceived job insecurity. Job insecurity is defined as “a personal concern about the future of the job.” Such concern has been linked to having a negative influence on employees' work [9] and the general healthcare crisis [10]. An important way in which an organization can have an impact is by providing social support for its employees. This highlights the potential role that social support can play in minimizing negative outcomes outside of work and in the workplace [11]. For employees experiencing the impact of E-government policies such as lockdown, it is important for the organization to provide social support for them. Thus, studies on interventions that can reduce the impact of E-government policy on employees' healthcare crises are necessary. The sustainable healthcare system consists of five main dimensions, including long-term strategic perspective and innovativeness, disease prevention and health promotion, quality, institutionalization of environmental concerns, and institutional accountability and individual responsibility (see Figure 1).

## 2. Theoretical Background and Hypothesis Development

Research suggests that job loss happens more frequently and those with employment become uncertain about the future of the job as job insecurity rises [12]. Job insecurity is a stressful experience that research has documented to be related to negative feelings and distress [13, 14]. Given the rarity of the COVID-19 pandemic, limited studies have investigated the possible psychological implications of job insecurity [15]. However, some evidence has shown a significant mental health burden caused by job insecurity due to the COVID-19 pandemic. Such a conclusion is consistent with prior research that demonstrated the negative mental health impacts of job insecurity before the current pandemic [16, 17]. Recent research concerning the COVID-19 pandemic reported that job insecurity is related to healthcare crises [18].

Healthcare crises is defined as the “experience of feeling good and/or feeling authentic and meaningful in one's life” [19]. This definition takes into consideration the eudaimonic and hedonic dimensions of healthcare crises; the formal pertains to the accomplishment of an individual's potential and a meaningful life; the latter is concerned with the absence of negative affect and the presence of negative affect. Analysis of healthcare crises in the workplace has focused on job characteristics and work-family conflict [20, 21]. Therefore, more research needs to be conducted during the COVID-19 pandemic.

Social support is the “experience that one is cared for, esteemed, and a part of a mutually supportive social network” [22]. Research has documented the advantageous impacts on mental and physical health [22]. Several studies have given social support a central role in reducing distress in the workplace [23, 24]. House [25] suggested that social support impacts stress and its associated outcomes in three distinctive ways. Firstly, social support could have a direct influence on outcomes in such a manner that individuals who experience greater levels of support are expected to have less dissatisfaction with their jobs and better health. Secondly, it could have a main or direct impact on perceived stress such that when social support is present, the degree of stress perceived is minimized. Lastly, the third effect is buffering. The focal point here is that social support could change the relationship between stress and its outcomes. The latter aligns with the objective of our study to test if the indirect effect of E-government policy on healthcare crises is contingent on social support.

### 2.1. E-Government Policy and Healthcare Crises

E-government policies such as restrictions have been reported to have an adversarial effect on healthcare crises [26–28]. While E-government policies such as restrictions are intended to curb the spread of the disease, they have rapidly changed the very fabric of human existence, restricting or even forbidding any forms of social interactions and requiring people to rapidly adapt to entirely different routines. From this standpoint, Rudolph and Zacher [29] pointed out that even though these E-government measures are effective in reducing the spread of viruses, they are psychological stressors, in other words. Some countries put in place partial lockdowns, while some introduced full lockdowns and others introduced quarantines. Such measures lead to restrictions to varying degrees on many parts of their population. Prior studies have found such measures to have a detrimental effect on healthcare crises and general physical health [30]. This study was conducted within the western context and outside the tourism industry. Thus, the relationship between E-government policy and healthcare crises in the domain of the tourism industry, particularly in Iraq, has not yet been explored. Given the above evidence and advancing the existing literature, we hypothesize the following:

H1: E-government policy is significantly associated with healthcare crises.

### 2.2. E-Government Policy and Job Insecurity

Researchers from all across the world have been drawn to the Learning Healthcare System model. Large-scale health data reuse and the incorporation of patient perspectives into care models can result in individualized treatment, lower healthcare costs, and less resource consumption [31, 32]. In recent history, the potential consequences and associated impacts related to COVID-19 measures are unprecedented [33]. Individuals are also said to be poor predictors of their own future effects [34, 35]. From this standpoint, Greenhalgh and Rosenblatt [36] described job insecurity as the fear that an employee faces while working in an organization with a threat of employment. Thus, the relationship between E-government policy and job insecurity could be particularly important during the time of the COVID-19 pandemic. In addition, while governments provide financial support for businesses, the implementation of a nationwide lockdown disrupts business activities, and such disruption would cause employees to fear for the future of their jobs. Based on the above reasoning, we hypothesize the following:

H2: E-government policy is negatively associated with job insecurity.

### 2.3. Job Insecurity and Healthcare Crises

Job insecurity was linked to both mental health complaints (e.g., emotional exhaustion, depressive feelings, anxiety, somatic symptoms, social dysfunction, and irritation) and physical health complaints (e.g., headaches, stress, increased blood pressure, and sleeping disorders) [37–40]. Further, Khan et al. [4] mentioned that job insecurity is one of the important factors that lead to restlessness among employees, thus affecting their healthcare crises. Similarly, Llosa et al. [41] concluded that job insecurity significantly affects employees' mental health. When it comes to the COVID-19 pandemic, job insecurity could be a particularly important issue. The economic decline during the pandemic is likely to heighten job insecurity among employees because organizations are prone to suffering more economic losses. Therefore, in the pandemic context, more research needs to be carried out, especially in the tourism industry, on the effect of insecurity on healthcare crises by taking the dynamic nature of the situation into account. Given the above evidence, we posit the following:

H3: Job insecurity has a negative effect on healthcare crises.

### 2.4. The Mediating Role of Job Insecurity

Meyer et al. [42] described job insecurity as “a perceived threat to the continuity and stability of employment as it is currently experienced.” Moreover, several studies accept that the fear of job loss can worsen the mental healthcare crises during a pandemic [43, 44], and policymakers must be aware that E-government measures during a pandemic come with significant welfare effects [14, 45]. Zhang et al. [8] reported that one month into the pandemic, in a Chinese sample, healthcare crises of those that were very physically active before the onset of the disease were specifically sensitive to the severity of the disease in their vicinity. From this standpoint, a cross-national study of 27 European countries on actual and expected employment losses found that job insecurity is associated with several aspects of physical and mental health [46]. Similarly, the study of Llosa et al. [41] concluded that having low satisfaction with life among employees, together with other psychological and mental issues, is common among employees who perceive that their employment is not secure. Previous research has stressed that job security has several detrimental effects. Kalleberg [47] identified complaints regarding low job satisfaction, lack of commitment, and mental health as a few of the adversarial effects of job insecurity. In this context, we are proposing that job insecurity mediates the relationship between E-government policy and healthcare crises. Thus, we posit the following:

H4: Job insecurity mediates the relationship between E-government policy and healthcare crises.

### 2.5. The Moderating Effect of Social Support

Social support measures individuals' perceptions pertaining to the general availability of support or satisfaction with support provided [48]. The pandemic is a global menace. Highly contagious viruses such as COVID-19 afflict the mental health of people since they affect the healthcare crises of people (8). Related studies have shown that individuals with low social support are more likely to experience emotional strain during the pandemic [42]. The study concluded that social support (at home and at work) moderated the relationship between pandemic duration and psychological healthcare crises across groups and recommended that interventions should be aimed at minimizing the psychological side-effects of the pandemic for the working class.

The current healthcare system infrastructure is still insufficient to deal with the rising number of COVID-19 cases, which has also revealed the healthcare system's low capacity to manage medical waste. Stuart and Adams [49] tried to foster the debate about reforming the Canadian healthcare system by adapting Maslow's hierarchy of needs to the context of healthcare sustainability (see Figure 2). The COVID-19 pandemic has highlighted the flaws in the patient referral system as well as the healthcare sector's poor ability to provide crucial health services during long-term emergencies. The Indonesian government must improve the country's healthcare infrastructure. A variety of techniques have been offered to address these rising issues. Despite this, the difficulties of improving healthcare capacity underline the fact that such efforts may only be one component of the pandemic response equation. Effective pandemic response requires governments to commit to increasing healthcare capacity while also flattening the curve (family and friend support) in moderating stress and its outcomes. Thus, we posit the following:

H5: Social support moderates the relationship between the E-government policy and healthcare crises in a manner that higher social support reduces the negative effect of E-government policy on healthcare crises.

## 3. Method

The participants in this study were full-time employees of 51 tourist destinations from different provinces in Iraq. These tourist destinations are very important to the national economy because people visit them from all over the world for religious activities. The tourist destinations surveyed include Imam Hussain's Shrine, Al Abbas Holy Shrine, Tal Al Zainabeiah site, Al Yassin Mosque, Al Sahlah Great Mosque, Imam Ali Mosque, etc. A self-reported questionnaire survey was sent out to the participants to assess our study variable. Before data collection, human resource (HR) managers of these tourist centers were contacted to seek their permission. After explaining the purpose of our study to them, employees were encouraged to participate in our study, and we assured them that their anonymity and confidentiality would be protected. Voluntary participation was sought, so a purposeful sampling method was employed in this study, and no monetary incentives were given to the participants. The questionnaire was sent using Google Forms. While some participants returned the completed questionnaires immediately, some took 24 hours to return the completed survey. The data was gathered between April 12 and July 2, 2020.

A total of 650 questionnaires were administered, of which 435 valid responses were recovered. A total of 215 invalid responses were removed. Following the removal of invalid responses, we obtained a 66.92% response rate. Please refer to Table 1 for demographic characteristics. The final sample consists of 292 males (67.13%) and 143 females (32.87%). About 92% of the participants were over the age of 28, and the majority (91%) had at least a university degree. Of those, 375 (86.20%) had at least 6 years of work experience.

## 4. Measures

Table 2 presents the descriptive statistics and Pearson's correlation values between all variables of the study. The results of the correlations to each variable are discussed separately in this section.

### 4.1. E-Government Policy

The public's perceptions of important responsibilities of the E-government in relation to the pandemic were measured using eight items. The first five items were sourced from Lazarus et al., while the latter three were sourced from the WHO [50]. The 8 items were graded on a 5-point Likert scale, with 1 representing “totally disagree” and 5 representing “absolutely agree.” This scale has been validated in a recent study [51]. The measure has great reliability in this study (Cronbach′s alpha = 0.922).

### 4.2. Social Support

Social support was measured with six items. The first four items were taken from Eisenberger et al. [52] and two from Heaney [53]. The items measure the social support provided by the organization and supervisor. Employees were asked to state their disagreement or agreement (1 = strongly disagree to 5 = strongly agree). The scale has reliability (Cronbach′s alpha = 0.931).

### 4.3. Job Insecurity

Job security measures employees' concerns about their job. Four items about perceived job insecurity were adopted from De Witte et al. [10]. The items include “Chances are I will soon lose my job” and “I feel insecure about the future of my job.” Participants rated each item on a 5-point Likert scale from 1 (“totally disagree”) to “5”, (“totally agree”). In the present study, this scale has reliability (Cronbach′s alpha = 0.897).

### 4.4. Healthcare Crises

Healthcare crises were measured with 5 items. The items were taken from Bech et al. [54]. The items were used to assess the mental health crises of the participants in the past 1 month. The sample items were worded positively, and they included “I have felt calm and relaxed” and “I have felt cheerful and in good spirits.” In this study, Cronbach's alpha was 0.81.

## 5. Analysis and Results

SPSS 27.0 and AMOS 24.0 were used for data collection and analysis. SPSS was used to analyse the demographic information, descriptive statistics (mean and standard deviation), and correlation (relationship between constructs). AMOS was used for construct validity and reliability. This present study chose PROCESS macro in SPSS overstructural equation modelling (SEM) to verify our study's hypotheses. The reason for this is that, in contrast to the SEM program, conditional indirect effects and moderation-mediation indices can be computed in a simple and effective manner, thus to avoid the issues caused by interaction estimation in the latent variable method [55].

### 5.1. Measurement Model

The measurement model was evaluated using Henseler et al. [56] standards, which included Cronbach's alpha, convergent validity, and discriminant validity. Cronbach's alpha () and composite reliability (CR) values were higher than the criteria level of 0.70, as shown in Table 3. Furthermore, in this investigation, the AVE for all observed variables was greater than 0.50. As a result, the findings demonstrate high reliability and convergent validity (p. 4).

The public's trust is built on the promise of net benefits. The public's faith in the healthcare system legitimizes the system's operations and encourages the public to participate in healthcare-related activities. Furthermore, high or low levels of public confidence in other sections of the government system have spillover effects on public trust levels. Finally, various players both within and outside the healthcare system have an impact on public trust. This conceptual framework will need to be translated into policy guidelines and a measurement scale in the future, as well as validated for healthcare systems other than the British NHS.

Table 4 demonstrates the discriminant validity where the square root of the AVEs of each latent variable should be greater than the surrounding correlations. As illustrated in Table 4, each of the square roots in the diagonal is greater than the surrounding correlation, thereby showing further proof of discriminant validity [57].

### 5.2. Common Method Bias

Harman's one single factor was applied to deal with the possibility of common method bias [58]. When all the measurement items were loaded, the first factor explained 38.29% of all the four factors with values greater than one. This is less than the acceptable value of 50%. Thus, indicating common method bias is not a concern in this study. In addition, the variance inflation factor (VIF) values for correlation between all observed variables in this study were below 4, suggesting no multicollinearity clouded our results [59].

### 5.3. Testing for Direct and Mediation Effects

As demonstrated in Table 4, the results of a simple mediation model showed that E-government policy was significantly associated with healthcare crises (*B* = 1.01, *p* 0.001), supporting hypothesis H1. E-government policy was negatively associated with job insecurity (*B* = −0.928, *p* 0.001), supporting hypothesis H2. Job insecurity was negatively associated with healthcare crises while controlling for E-government policy (*B* = −0.289, *p* 0.001), validating hypothesis H3. Finally, the result of the bias-corrected percentile bootstrap method showed that the indirect effect path between E-government policy and healthcare crises via job insecurity was statistically significant, as shown in Table 5 (*B* = −0.217, SE = 0.072, 95% CI = −0.421, -0.107), lying outside zero, validating hypothesis H4. The indirect effect (mediation) explained 41.25% of the total effect. Furthermore, the four conditions satisfied Mackinnon's four-step procedure (41) and supported the mediating effect.

### 5.4. Moderated Mediation

The results revealed that social support is a moderator of the indirect effect of E-government policy on healthcare crises. The plot indicated that the presence of high social support would reduce the negative impact of E-government policy on job insecurity compared to low social support and high job insecurity.

The conditional indirect effect of social E-government support on healthcare crises through job insecurity at the values of social support was analysed when the scores of social support were the sample mean (±SD). The results show that the three conditional indirect effects were all statistically significant, and bootstrap confidence intervals validated these results (see Table 6).

In summary, the results supported a moderated mediated model where job insecurity was the partial mediator of the impact of E-government policy on healthcare crises.

## 6. Discussion

This study examined the impact of E-government policy and healthcare crises during COVID-19. First, E-government policy was found to be a significant predictor of employees' healthcare crises. This result is consistent with prior research [1, 2]. The consistency of this pattern of results suggests that E-government measures during the COVID-19 pandemic affect employees' healthcare crises. For example, Khan et al. [4] suggested that the E-government ignored psychological aspects associated with mental health. For this reason, an E-government program should include measures to improve employees' healthcare crises. Second, the results revealed that E-government policy negatively predicted job insecurity. This aligns with the conclusion of [31, 32]. The observation here is that E-government policies such as lockdown have left employees anxious and worried about whether they will keep their job or not, which is not entirely in their control. Third, job insecurity negatively and significantly predicted healthcare crises. This result is in line with prior research [38]. The discovery of a negative relationship between job insecurity and healthcare crises in the context of the tourism industry in Iraq shows that such a relationship is not limited to the western context only.

Lastly, the moderated mediation results showed a significant direct effect of E-government policy and a significant indirect effect of E-government policy on job insecurity. This means the effect of E-government policy on healthcare crises is partly mediated by job insecurity (see Table 7). The observation here is that employees who received low social support from their organizations are prone to experiencing higher job insecurity, while those who received higher social support will experience lower job insecurity, implying the degree of protection is dependent upon the level of social support. Thus, it provides support for [11].

### 6.1. Theoretical Implications

The current research tested a moderated mediation model using samples from 51 tourist destinations where we hypothesized that the impact of E-government policy on healthcare crises would be mediated by job insecurity. The indirect effects of E-government policy on healthcare crises through job insecurity were then moderated by the levels of social support. Our findings contribute in several ways to the limited knowledge of E-government policy and employees' healthcare crises in the context of the pandemic, particularly in the tourism sector in Iraq.

First, the results of this contribute to research on healthcare crises by investigating the impact of macro-level factor such as E-government policy on healthcare crises of employees in the tourism sector. Second, to our knowledge, this is the first that investigated the impact of E-government policy on healthcare crises through the mediating effect of job insecurity and also if the indirect effect is contingent on social support. Third, this study is unique in testing social support as the moderator that can provide intuition for establishing organization-employee social support during the pandemic.

### 6.2. Practical and Managerial Implications

Our study has several practical implications. Firstly, this research has the potential to assist organizations by advising them on how to manage their employees during a crisis. It emphasizes the need for management to give importance to psychological aspects by providing employees with measures that can promote their healthcare crisis. In the tourism industry, healthcare crises of employees should be given priority because customers interact with employees to provide them with services.

Second, as a result of the abrupt changes in the way humans live due to the pandemic, this study might help organizations develop strategies that can provide or improve social support for their employees. For example, human resource managers should focus on ways to avoid job insecurity through the implementation of educational programs to improve social support. Thus, employers may play an important role by giving employees regular and accurate information during the pandemic to diffuse rumors and diminish any individual suspicions and concerns.

## 7. Conclusion

Generally speaking, this empirical study examines the E-government policy on healthcare crises from an employee's perspective. A self-reported measure was used to collect the data, and the results revealed that E-government policy was a significant predictor of healthcare crises. Additionally, job insecurity was a critical mediator between E-government policy and healthcare crises, and social support was a critical moderator; employees with lower social support from their organization would experience higher job insecurity, and employees with higher social support experienced lower job insecurity. Furthermore, theoretical and managerial implications are discussed.

### 7.1. Limitations and Further Research

Despite the achievement of this study, the present study is not without limitations that future studies should take into consideration. Firstly, the sample was limited to the tourism industry of Iraq, so generalization to other sectors and other countries is required in future studies. Secondly, our study used a cross-sectional design, which only permits inferring relationships between variables but not potential causality or directions of the relationships. The data collected was based on the immediate impact of the COVID-19 pandemic at the time of collection. Therefore, because the self-reporting method was used to measure E-government policy, job insecurity, social support, and healthcare crises, the participants could respond in a way that fit their social desirability bias [58]. Future research should use more objective and measurement tools (longitudinal research design) to confirm the consistency of our results. Thirdly, we did not control for all variables that might have affected the results, for example, gender and age. Future studies could benefit from taking demographic information into consideration. Finally, future studies could go a bit further beyond this research by testing whether the relationship between E-government policy and healthcare crises is also moderated by social support.

## Figures and Tables

**Figure 1:** Dimensions of healthcare system sustainability.

**Figure 2:** Pyramid of healthcare needs [49].

**Table 1:** Characteristics of survey participants.

Demographic information (*N* = 435)	Frequency	Percentage (%)
Gender	
Male	292	67.13
Female	143	32.87
Age (years)		
18-27	12	2.76
28-37	112	25.75
38-47	242	55.63
48-57	57	13.10
58 and over	12	2.76
Education		
High school	36	8.28
University first degree	333	76.55
Master degree	57	13.10
PhD degree	9	2.07
Experience (years)		
1-5 years	60	13.79
6-10 years	112	25.75
11-15 years	203	46.67
More than 15 years	60	13.79

**Table 2:** Descriptive statistics and Pearson's correlation.

Variables	M	SD	GP	SS	JI	HC
GP	3.767	0.529	(0.793)			
SS	3.132	0.667	0.563^∗∗^	(0.794)		
JI	3.447	0.596	-0.611^∗∗^	-0.499^∗∗^	(0.825)	
HC	4.137	0.582	0.459^∗∗^	0.821^∗∗^	-0.518^∗∗^	(0.775)

M: mean; SD: standard deviation. ^∗∗^Correlations are significant at the 0.01 level (2-tailed).

**Table 3:** Reliability and validity measure.

Variables	Measurement items	SFL	AVE	CR
E-government policy	GP1	0.642	0.629	0.929
	GP2	0.947		
	GP3	0.922		
	GP4	0.678		
	GP5	0.822		
	GP6	0.788		
	GP7	0.911		
	GP8	0.701		

Social support	SS1	0.926	0.631	0.948
	SS2	0.601		
	SS3	0.946		
	SS4	0.817		
	SS5	0.749		
	SS6	0.964		

Job insecurity	JI1	0.719	0.682	0.963
	JI2	0.829		
	JI3	0.841		
	JI4	0.906		

Healthcare crises	HC1	0.721	0.602	0.940
	HC2	0.852		
	HC3	0.760		
	HC4	0.827		
	HC5	0.838		

**Table 4:** Regression results for simple mediation.

	*B*	SE	*p*
Healthcare crises regressed on E-government policy	1.011	0.201	*p* ≤ 0.001
Job insecurity regressed on E-government policy	-0.928	0.194	*p* ≤ 0.001
Healthcare crises regressed on job insecurity, controlling for E-government policy	-0.289	0.039	*p* ≤ 0.001
Healthcare crises regressed on E-government policy, controlling for job insecurity	0.200	0.034	*p* ≤ 0.001

**Table 5:** Bootstrap indirect effect of E-government policy on healthcare crises through Job Security.

	*B*	SE	LLCI	ULCI
Job insecurity	-0.217	0.072	-0.421	-0.107

**Table 6:** Regression results for conditional process analysis (*N* = 435).

	*B*	SE	*p*	LLCI	ULCI
Job insecurity					
E-government policy (GP)	-0.247	0.039	*p* ≤ 0.001	-0.169	-0.325
Social support (SS)	0.146	0.021	*p* ≤ 0.001	0.184	0.308
GP x SS	-0.101	0.052	0.032	-0.208	-0.001
Healthcare crises					
E-government policy	0.200	0.039	*p* ≤ 0.001	0.123	0.277
Job insecurity	-0.289	0.034	*p* ≤ 0.001	-0.221	0.019
Conditional indirect effect at specified value of social support					
1 SD below the mean	0.314	0.053	*p* ≤ 0.001	0.210	0.419
Mean	0.247	0.039	*p* ≤ 0.001	0.169	0.325
1 SD above the mean	0.179	0.059	0.007	0.075	0.283

**Table 7:** Index of moderated mediation.

	Index	SE	LLCI	ULCI
Social support	0.029	0.017	0.065	0.194

## Data Availability

Data are available upon request.
